# Biodiversity of Gut Microbiota: Impact of Various Host and Environmental Factors

**DOI:** 10.1155/2021/5575245

**Published:** 2021-05-12

**Authors:** Haseeb Anwar, Arslan Iftikhar, Humaira Muzaffar, Ahmad Almatroudi, Khaled S. Allemailem, Soha Navaid, Sana Saleem, Mohsin Khurshid

**Affiliations:** ^1^Department of Physiology, Government College University, Faisalabad, Pakistan; ^2^Department of Medical Laboratories, College of Applied Medical Sciences, Qassim University, Buraydah, Saudi Arabia; ^3^Department of Microbiology, Government College University, Faisalabad, Pakistan

## Abstract

Human bodies encompass very important symbiotic and mutualistic relationships with tiny creatures known as microbiota. Trillions of these tiny creatures including protozoa, viruses, bacteria, and fungi are present in and on our bodies. They play important roles in various physiological mechanisms of our bodies. In return, our bodies provide them with the habitat and food necessary for their survival. In this review, we comprehend the gut microbial species present in various regions of the gut. We can get benefits from microbiota only if they are present in appropriate concentrations, as if their concentration is altered, it will lead to dysbiosis of microbiota which further contributes to various health ailments. The composition, diversity, and functionality of gut microbiota do not remain static throughout life as they keep on changing over time. In this review, we also reviewed the various biotic and abiotic factors influencing the quantity and quality of these microbiota. These factors serve a significant role in shaping the gut microbiota population.

## 1. Background

It is interesting to know that there are tiny creatures that reside in our bodies as a result of a symbiotic relationship between them and ourselves [1]. We provide them with a habitat where they can live and also provide them with food on which they feed upon, and in return, they benefit us in so many ways by interacting with various physiological phenomena going on in our bodies. These tiny creatures that live on and inside our bodies are termed as microbes (bacteria, fungi, protozoa, and viruses) [2]. Microbiota and microbiome are two important terms related to microbes. Microbiota refers to the microbial communities which inhabit a particular habitat while microbiome refers to the collective genome of all the microbial cells which reside in the human body [3]. The human microbiota is the collection of trillions of microbes living in and on the human body [4]. These microbes inhabit various body organs including the mouth, gut, reproductive organs, and on the skin.

In the literature archive, the therapeutic potential of these microbiota has been linked to the diagnosis, management, and treatment of various disorders [5]. They have been associated with the prevention and progression of various central nervous system disorders like multiple sclerosis [6, 7]. They have also been linked to the prevention and treatment of cardiovascular diseases like hypertension [8, 9], along with enhanced predisposition towards various viral and bacterial infections. In various other studies, these “healthy” microbiota have been associated with the treatment of various metabolic diseases like obesity [10, 11], diabetes, and nonalcoholic fatty liver disease (NAFLD) [12]. The emerging role of these microbiota has also been reported as a mitigation strategy against various respiratory viral infections [13] including COVID-19 [14, 15]. The colonization and distribution of various intestinal microbiota at particular sites in the gut, their disturbance, and associated intestinal immune disorders have been linked to the elicitation of various tumors [16, 17] as well. In this review, we evaluated the various biotic and abiotic factors affecting the quantity and quality of microbiota. These factors play important roles in molding the gut microbiota population.

## 2. Gut Microbiota Composition

A vast habitat of microbes residing in the human body lies in the gut known as the gut microbiome. It is estimated that there are about 100 trillion microbes present in our gastrointestinal tract that are mainly comprised of bacteria along with other microbes like fungi, protozoa, and viruses. Initially, it was thought that there are 10 times more microbial cells than the human cells residing in our body [18], but now, a recent insight has given us an idea that human cells and microbial cells are present in our body in 1 : 1 which depicts the fact that there are approximately equal microbial and human cells [19]. Our genome comprises about 23,000 genes, while, on the contrary, the microbiome comprises around 3 million genes [20]. The microbes present in the gut are in increasing concentrations from the stomach to the colon, which means that the microbial population in both concentration and diversity is high in the last portions of the intestine, i.e., colon/large intestine [21]. It is estimated that the microbial mass starts from 10^2^ (stomach) to 10^14^ (colon) which is a huge difference indeed [22]. The Human Microbiome Project has provided comprehensive data about gut microbiome on 2172 species isolated from human beings, classified into 12 different phyla, of which 93.5% belonged to *Proteobacteria*, *Firmicutes*, *Actinobacteria*, and *Bacteroidetes* [23]. Another study has coined that among gut microbes, thousands of bacterial species constitute in the human gut, and the most abundant genera include *Bacteroides*, *Clostridium*, *Fusobacterium*, *Eubacterium*, *Ruminococcus*, *Peptococcus*, *Peptostreptococcus*, *Lactobacillus*, and *Bifidobacterium* [24].

### 2.1. Gut Microbial Species in Various Regions of the Gut

When we ingest food, it firstly comes in contact with salivary glands which, during mastication, secrete amylases and lipases. After that, food goes to the stomach which retains the food for some period of time. In the stomach, which is the first and foremost region of the gastrointestinal tract, there is the least diversity of gut microbiota. Its reason could be the more acidic pH gradient, which the entire gut microflora could not tolerate [25]. Then, certain other digestive enzymes (proteases, lipases, and amylases) enter into the small intestine from the pancreas through the biliary duct. These digestive enzymes break down the food into simple sugars, amino acids, and fatty acids which are then absorbed from the small intestine into general circulation. Those food components which are not digested by host digestive enzymes are then moved forward towards the large intestine via the ileocecal valve. This ileocecal valve is crucial for maintaining a host-symbiotic relationship with gut microflora as it prevents the backflow of content from the large intestine to the small intestine [26]. Thus, it restricts most of the microbial mass of the gastrointestinal tract into the large intestine. The large intestine contains saccharolytic bacteria that can convert nondigestible food components like fibers, resistant starches, some peptides, and lipids which failed to be broken down by the host digestive enzymes. Gut microbiota can ferment nondigestible food components into short-chain fatty acids like butyrate [27]. The reasons why there is less population of gut microbiota residing in the stomach and small intestine are firstly acidic pH of gastric content [28], the bactericidal nature of bile acids which are secreted from the liver into the small intestine, increased peristalsis through the small intestine, the immunoglobulin IgA present in gut mucosa which act as an antimicrobial agent as it leads to the agglutination of microbiota [29], and furtherly the inability of most of the microbiota to stay longer in the small intestine due to peristalsis [30]. The microbial mass and the microbial species including both autochthonous and allochthonous [25] present in various regions of the gut are enlisted in Table 1. The term autochthonous describes the microflora that is present endogenously and is commonly present in almost all the hosts whereas the term allochthonous describes those species of microbiota that are derived from exogenous sources and are not common to every host but can be present in more than one host.

## 3. Modulatory Factors of Gut Microbiota

There are so many factors including geographical distribution, dietary interventions, use of probiotics and prebiotics, use of antibiotics, and environmental factors, like sanitary condition, air pollution, and disrupting chemicals, which serve as modulatory factors that ultimately influence the composition, diversity, and functionality of gut microbiome as shown in Table 2.

### 3.1. Effect of Geographical Distribution and Dietary Habits

We all live in different geographical regions, like some live in the East or some live in the West; due to these geographical distributions, our lifestyle varies which leads to variations in dietary habits, like some eat more vegetables just relying upon a fresh, leafy, and fibrous diet while some rely upon an only-protein diet, like they are more flesh lovers, or with the increase in modernization, we are more inclined towards junk food [31]. So, these variations also affect our gut microbiome in a way that increases the number of one species while reducing the other one just by fluctuations in dietary habits [32]. This phenomenon can be well understood by an example in that some bacterial species are vegetable lovers or their growth depends upon it, so when our diet contains more and more vegetables/fibers, then there will be a rise in such vegetable lover bacterial species as they feed upon it, while on the other hand, as the meat lover bacterial species may not find the substances upon which they can feed upon, their number will get diminished [33]. This phenomenon is reversible which sounds pretty good in that if someone wants to modify his gut microbiome, he can do it easily by shifting the dietary patterns. Thus, we can say that we are responsible for our gut microbiome as we have entered an era where we can fully understand that we are now able to modify our health patterns via food or our dietary habits, and ultimately, we can measure its side effects and beneficial effects just by looking at our gut microbiome. This phenomenon is also proven by various studies. For example, the *Bacteroides* genus is highly associated with the consumption of animal proteins, amino acids, and saturated fats, which are typical components of the western diet, while the *Prevotella* genus is associated with the consumption of carbohydrates and simple sugars, which are typical of agrarian societies [34]. People with a *Bacteroides*-dominated gut microbiome will gain a *Prevotella*-dominated microbiome by switching from a western diet to a carbohydrate-based diet for an extended period of time [35] Table 3.

### 3.2. Effect of Different Stages of Life

Other than geographical distribution and dietary habits, another factor that influences the gut microbiota is age. Children, adults, and elderly people have different sorts of gut microbiome as shown in Figure 1.

#### 3.2.1. Gut Microbiota during Prenatal Development

Amniotic fluid and placenta are the first sites where the gut microbiota starts to evolve [36]. The microbiota is transferred to the fetus from the maternal blood via meconium [37], amniotic fluid [38], and placenta [39]. That was confirmed by orally administering some labeled species of bacteria, like *Enterococcus faecium* to the mother during her period of gestation [40], and after that, stool samples of the newborn were analyzed which showed the presence of the labeled bacterial species which confirmed that microbiota is transferred from mother to fetus in in utero life span [41].

#### 3.2.2. Gut Microbiota at Birth Stage

Then further, the microbiota is shaped based on delivery patterns. The children who are born vaginally have the prevalence of *Prevotella* and *Lactobacillus* bacteria in the infant's gut [42], which are colonized from the vagina of their mother.

The children who are born through C-section/cesarean delivery have dominated gut bacterial species of *Streptococcus*, *Corynebacterium*, and *Propionibacterium* which are derived from the skin of that mother. At the time of birth, the evolution of microbiota is termed as primary microbiota which evolves to become more diverse [43].

#### 3.2.3. Gut Microbiota during Infancy and Toddlerhood

The feeding pattern of neonates and infants make the interindividuals' differences higher in children than in adults. These interindividual differences in children are due to a specific reason that some neonates are fed with breastfeeding milk and some are dependent upon formula feeds [44]; these variations of feeding patterns lead to diversity and variations in gut microbiota composition. In infants who are given mother feed (breast-fed infants) are dominant with *Lactobacillus* and *Bifidobacterium* [45] in their gut while formula-fed infants have dominant species of *Enterococcus*, *Bacteroides*, *Streptococcus*, *Clostridia*, and *Enterobacteria* [46].

#### 3.2.4. Gut Microbiota during Adult Stage

One study was done in which bacterial species of fecal samples from individuals of different age groups (0-70 years) were collected. Their study depicted the results in such a way that diversity of gut microbiota was significantly higher in adults than in children while the interindividual differences were higher in children than in adults [42]. The composition of gut microbiota turns into an adult-like pattern after 3 years of life [31].

### 3.3. Effect of Dietary Interventions

We have a symbiotic mutualistic relationship with our microbiota which means that we provide them with habitat for their living, and also, we provide them with food. The food which we ingest is also utilized by gut microbiota, and our dietary patterns allow shaping the composition and dominance of certain microbial species residing in the gut. For instance, consumption of diet containing high saturated fatty acids and high protein content can cause gut dysbiosis which has been linked to pathogenies of various ailments including autoimmune diseases, central nervous system disorders, and various infections [47].

### 3.4. Effect of Probiotics

The food we eat has a significantly vital role on the gut microbiota. The probiotic which we ingest as live bacteria in the form of food supplements has a positive impact on our gut microbiome as its usage provides beneficial integrity to the gut microbiome [55]. The most important strains of bacteria which are considered probiotics are *Lactobacillus*, which is in the *Firmicutes* group, and *Bifidobacterium*, a type of *Actinobacteria* [56]. Both are commonly found in foods that are labeled as containing probiotics. Probiotics are also found in dietary supplements and are added to foods and beverages such as protein shakes, fermented dairy products as well as dietary supplements, and fruit juice [57]. The genus *Bifidobacterium* has some strains of bacterial species which can produce short-chain fatty acids, like acetate and lactate. These short-chain fatty acids have a positive and beneficial impact on the gastrointestinal tract by having a direct impact or by having an indirect effect by further converting via other gut microbes into other short-chain fatty acids, like butyrate [58]. Probiotics are now fundamentally used in the form of food or dietary supplements. Probiotics perform their function by manipulating the gut microflora, by suppressing the growth of disease-causing pathogenic microbes, inducing fortification of the intestinal epithelial barrier, by stimulating epithelial cell proliferation and differentiation. Probiotics mostly perform their function by inducing the host immune system to produce *β*-defensin and immunoglobulin A (IgA), thus manipulating the gut microflora and suppressing the growth of pathogenic bacteria [59]. Probiotics help in fortifying the intestinal epithelium by maintaining the tight junctions and also help in the production of mucin by intestinal epithelial cells. Probiotic-mediated immunomodulation occurs via secretion of cytokines which can also affect proliferation and differentiation of immune cells [60] and T cells and also help in proliferation of intestinal epithelial cells [61].

### 3.5. Effect of Prebiotics

Prebiotics are considered as food for bacteria. Naturally occurring prebiotics are found in foods that are rich in fiber content like vegetables, fruits, whole grains, and legumes like peas and beans [62]. Some synthetic prebiotics include inulin, and oligosaccharides are also available. Prebiotics are most often found in foods that are rich in fiber content [61]. Fiber-containing foods should be incorporated into a daily diet as it is recommended to take 25-38 grams of fiber per day. Gut microbiota utilizes these ingested fibers by metabolizing them into short-chain fatty acids, butyrate, propionate, and acetate [63]. These short-chain fatty acids modulate the gastrointestinal tract in so many ways. Short-chain fatty acids provide relief in constipation and diarrhea [64], help in absorption of calcium from intestinal cells into blood circulation, help in reducing the risk of colorectal cancer, and also nourish the cells present in the intestinal lining [65].

### 3.6. Effect of Antibiotics

Together with every scientific invention or discovery, there are some precautions in the usage associated with that discovery which have to be followed at any cost; otherwise, aside from giving or providing benefit, it will produce havoc. On the one side, the discovery of antibiotics brought upon a revolutionary change in curing the fatal diseases like tuberculosis and meningitis, which are caused by bacteria, but on the other side, their excessive usage has created antibiotic resistance in many bacterial strains [66].

The working mechanism of antibiotics occurs in three different ways. Firstly, by interfering with the synthesis of the bacterial cell wall because if there is no proper cell wall development, bacteria will not divide. When there is no division, there will be no multiplication. So, automatically, the bacterial community will get reduced in that particular site where the antibiotic has done its action [67]. Secondly, antibiotics interfere with the synthesis of proteins which are essential for bacterial cell survival like for reproduction or the synthesis of the bacterial cell wall, or the processing of nutrients. Thirdly, they deliberately destroy bacterial DNA to reduce the ability of bacteria to divide further.

The excessive use of antibiotic drugs, more specifically the over usage of broad-spectrum antibiotics, has rendered the bacteria to develop resistance against most of the antibiotics. There are different ways by which bacteria develop antibiotic resistance, either by causing bacterial cell wall impermeability by which antibiotic molecules will not get any entry into the bacterial cell, by modifying the binding region or site due to which antibiotics are not able to bind to bacterial regions required for the antibiotic to perform its antibacterial action, by inactivating the antibiotic by adding a phosphate group to the antibiotic molecule to lessen its ability to get attached to the bacterial ribosomes, or by causing an efflux of dug immediately when it got entry inside the bacterial cell [68]. These are the resistance mechanisms that bacteria apply to cause antibiotic resistance when there is excessive usage of antibiotics. These resistance mechanisms are incorporated into bacterial genes present in bacterial DNA. We know reproduction is the mechanism that causes the transmission of those traits which reside in our genes, so in bacteria, during their multiplication, they also transmit these resistance mechanisms against antibiotics. If the mating occurs in those bacterial strains having resistance genes against two bacterial strains or having resistance genes against two different antibiotics, then there will be the formation of “superbugs” with various resistances against several antibiotics [69].

Thus, there is an interplay between microbes (gut microbiota) and medicines as antibiotics disrupt the natural microbiota in a way that these drugs not only kill the harmful disease-causing bacteria but also may interfere with the disruption of natural microbiota, thus leading to infectious diseases and other various digestive issues. Gut microbiota can also have the ability to modify some of the drugs during metabolism. So, the metabolic end products of these drugs may interfere with the normal composition of microbiota by causing severe side effects.

If we use ciprofloxacin against urinary tract infection, it will not only attack the targeted bacteria like *E. coli* that is only present in the urinary tract; rather, this antibiotic will sweep off its targeted bacteria from all the sites where it traveled through to reach its target [70]. Moreover, ciprofloxacin is a broad-spectrum antibiotic that can target most of the gram-negative and many of the gram-positive bacteria residing in different locations of our body. If we do an antibiotic course for 3-5 days, then two phenomena will occur; firstly, the targeted bacteria will develop resistance against that antibiotic. So, most of the bacteria will become resistant commensals, start to share their resistance genes, and become superbugs. Secondly, with the continuous usage of that antibiotic, most of the nonresistant commensal bacteria will be swept out from the body. The health ailment associated with the excessive usage of antibiotics is that they sweep out the essential/good bacteria along with the targeted bacteria and disrupt this balance, so if some bacterial invasions may come during this period, there will be no further defending bacterial strains to compete.

### 3.7. Effect of Air Pollution

With the increase in the advent of modernization in the form of urbanization, the public health concern is also increasing day by day. Various health ailments are going to increase with the increase in air pollution. The burden of various diseases is at its peak due to a rise in air pollution. A few years ago, it was considered that air pollution is only relevant to respiratory- and cardiovascular-related health disorders, but now, it is going to under hot discussion that air pollution also adversely affects our gastrointestinal tract by disrupting its gut microflora [71]. One may think how air pollution may result in deteriorating the gastrointestinal tract. The answer is simple: air pollution may get trapped in the food, and when we ingest this contaminated food, we may get affected.

Air pollution is termed as the presence of harmful substances in the air that can result from natural and human activities. Air pollution is a complex mixture of gases (which include ozone, carbon dioxide, sulfur dioxide, carbon monoxide, and nitrogen dioxide), particulate matter [72] that includes combustion of fossil fuels/car exhaust, polycyclic aromatic hydrocarbons/PAHS, pollens, spores, microbial particles, mineral dust, organic carbon, nitrates, and sulfate [73]. Atmospheric particulate matter and, above all, the air pollution are worldwide environmental problems, having several health ailments. Particulate matter is termed as the size of a particle whose diameter is in a range of 2.5 *μ*m-10 *μ*m [71]. The air pollution which comprises gases and particulate matter arises due to local sources, like emissions from factories, chimneys, livestock, and also fossil fuels [72].

The particulate matter and the ozone which are components of air pollution are now considered to have serious health ailments in a way that ozone and particulate matter increase the gut permeability, and also, they may destroy the tight junctions present in intestinal cell walls [74]. A little is known about the alterations which occur due to the effect of air pollution on gut microbiota. When the particulate matter is ingested, it is then metabolized by the gut microbiota into some other toxic metabolite which is detrimental for the whole gut, and if this metabolite comes into circulation, then it may cause some other effects. One study illustrated that gut microflora metabolized the inorganic arsenic which is a component of contaminated soils into toxic metabolites [75]. In another study, it was seen that gut microbiota converts the polycyclic aromatic hydrocarbon PAHs into those metabolites which mimic the activity of the estrogen hormone [76]. From these studies, we have come to know that our gut microbiota is involved in the bioactivation of inorganic compounds present in the particulate matter which is then proven to be dangerous in provoking various health ailments.

Recent advancements in biological studies have shown that air pollution is causing an alteration in the composition and physiology of the gut microbiota. Significant changes have been shown when particulate matter is mixed up with the feed of mice, where there are relative alterations that seem to occur in amounts of *Bacteroidetes*, *Firmicutes*, and *Verrucomicrobia* [77]. This dramatic shift in relative concentrations of gut microbiota results in the formation of branched-chain fatty acids (isobutyrate and isovalerate) which results in a decrease in the concentration of butyrate [78]. Butyrate is an essential fatty acid for the colonocytes and intestinal mucosal cells, and the reduction in butyrate will result in damage of the intestinal barrier and also lead to mucosal inflammation [79]. Another study has shown that when mice have been exposed to another pollutant, i.e., polychlorinated biphenyls (PCBs), the composition and metabolic processes associated with gut microbiota are also altered [80].

### 3.8. Effect of Disrupting Chemicals/Xenobiotics

Xenobiotics are substances that are foreign to the body. The word “xenobiotics” is derived from the Greek word “xenos,” meaning foreign, and “bios,” meaning life. Xenobiotics can come from natural resources (plant products, alkaloids) and from artificially manufactured sources (drugs, chemicals, and pesticides) [81]. It is now believed that a strong relationship is found between ingested chemicals and the gut microbiota in a way that the gut microbiota interacts with ingested environmental chemicals [82]. Recently, just like endocrine-disrupting chemicals, another term “microbiota-disrupting chemicals” has been coined [83]. The substances are considered as microbiota-disrupting chemicals which can modify the composition of microbiota or which can alter the activities of microbial community, and also, these alterations can cause serious health effects. Some food additives which are intentionally used to alter the microbiota composition for beneficial purposes will not be considered as gut microbiota disruptors as they do not cause any harm [84]. Therefore, to qualify as gut microbiota disruptors, it must cause a harmful health ailment by employing changes in the gut microbiota composition and functioning.

## 4. Conclusion

Gut microbiota is considered an “organ system” that carries out various vital functions in our bodies. Various factors are involved which interfere in the normal functioning of this vital organ system of the body which leads to microbial dysbiosis which not only alters the composition of microbial communities but also leads to alteration in normal physiological functioning associated with this normal microflora. In this review, we discussed various host and environmental factors that significantly influence the biodiversity of gut microbiota. We propose the scientific society to investigate various approaches to combat the modulatory factors to reduce the chances of gut microbial dysbiosis to keep this organ system intact both functionally and structurally.

## Figures and Tables

**Figure 1:** Various bacterial species residing in the gut in different stages of life.

**Table 1:** Microbial species in different regions of the gut.

	Region of the gut		
	Stomach	Small intestine (duodenum, jejunum, ileum)	Large intestine/colon
Microbial mass (cells/ml)	10^2-3^	10^3-4^, 10^4-5^, 10^8^	10^11-14^
Species present	Autochthonous: (i) *Helicobacter pylori*	Autochthonous: (i) *Enterococcus* (ii) *Bacteroides* (iii) *Ruminococcus* (iv) *Escherichia coli* (v) *Klebsiella* (vi) *Weissella* (vii) *Lactobacillus* (viii)*Clostridium* (ix) *Coprococcus*	Autochthonous: (i) *Firmicutes* (ii) *Bacteroidetes* (iii) *Actinobacteria* (iv) *Verrucomicrobia* (v) *Proteobacteria*
	Allochthonous: (i) *Fusobacterium* (ii) *Lactobacillus* (iii) *Neisseria* (iv) *Prevotella* (v) *Streptococcus*		
		Allochthonous: (i) *Streptococcus* (ii) *Lactobacillus*	

**Table 2:** Factors responsible for shaping gut microbiota in various stages of life.

Prenatal stage	Birth stage	Infancy stage	Adult stage
(i) Placenta (ii) Amniotic fluid (iii) Maternal stress (iv) Exposure to air pollution, PAHs, tobacco smoke, etc.	(i) Mode of delivery (vaginal delivery or caesarian delivery) (ii) Gestational age	(i) Feeding pattern (breastfed or formula-fed) (ii) Duration of lactation	(i) Dietary habits (ii) Lifestyle (iii) Use of antibiotics (iv) Exposure to environmental disruptors

**Table 3:** Composition and diversity of gut microbiota in different dietary contents.

	Phyla	Species	References
Diet rich in carbohydrates	Bacteroidetes	↑ *Prevotella enterotype*	[48]
	Firmicutes	↑ *Bifidobacteria* ↑ *Ruminococcus bromii* ↑ *Roseburia* groups	
	Actinobacteria	↑ *Bifidobacterium*	
Diet rich in fats	Bacteroidetes	↓ *Bacteroides spp.* ↓ *Rikenellaceae*	[49, 50]
	Proteobacteria	↓ *Desulfovibrio*	
	Firmicutes	↑ *Bacilli* ↑ *Roseburia spp.* ↑ *Erysipelotrichia* ↓ *Eubacterium rectale* ↓ *Ruminococcaceae*	
Diet rich in proteins	Bacteroidetes	↓ *Prevotella enterotype* ↑ *Bacteroides enterotype* ↑ *Bifidobacterium* ↑ *Lactobacillus* ↑ *Peptostreptococcus* ↑ *Rikinella*	[51, 52]
	Deferribacteres	↑ *Mucispirillum*	
	Proteobacteria	↑ *Desulfovibrio*	
	Firmicutes	↑ *Clostridium spp.*	
Diet rich in fibers	Bacteroidetes	↑ *Bacteroides spp.* ↑ *Prevotella spp.*	[53, 54]
	Actinobacteria	↑ *Bifidobacterium*	
	Proteobacteria	↓ *Desulfovibrio*	
	Firmicutes	↑ *Ruminococcus* ↑ *Lactobacillus* ↑ *Bacilli*	

## Abbreviations

IgA: Immunoglobulin A
PCBs: Polychlorinated biphenyls
PAHs: Polycyclic aromatic hydrocarbons.
